The article "Automatic Segmentation of Magnetic Resonance Images of Severe Patients with Advanced Liver Cancer and the Molecular Mechanism of Emodin-Induced Apoptosis of HepG2 Cells under the Deep Learning" was published in 2022. Journal: J Healthc Eng.

# Automatic Segmentation of Magnetic Resonance Images of Severe Patients with Advanced Liver Cancer and the Molecular Mechanism of Emodin-Induced Apoptosis of HepG2 Cells under the Deep Learning

**DOI:** 10.1155/2022/3951112

**Published:** 2022-03-07

**Authors:** Haiyan Zhao, Yuping Wang, Chen He, Jilin Yang, Yaoming Shi, Xiaolin Zhu

**Affiliations:** ^1^The Elderly of Treatment Department of Critical Medicine, The Frist Affiliated Hospital of Kunming Medical University, Kunming, Yunnan 650032, China; ^2^Undergraduate Clinical Major, Haiyuan College of Kunming Medical University, Kunming, Yunnan 65003, China

## Abstract

To improve the accuracy of clinical diagnosis of severe patients with advanced liver cancer and enhance the effect of chemotherapy treatment, the U-Net model was optimized by introducing the batch normalization (BN) layer and the dropout layer, and the segmentation training and verification of the optimized model were realized by the magnetic resonance (MR) image data. Subsequently, HepG2 cells were taken as the research objects and treated with 0, 10, 20, 40, 60, 80, and 100 *μ*mol/L emodin (EMO), respectively. The methyl thiazolyl tetrazolium (MTT) method was used to explore the changes in cell viability, the acridine orange (AO)/ethidium bromide (EB) and 4′,6-diamidino-2-phenylindole (DAPI) were used for staining, the Annexin V fluorescein isothiocyanate (FITC)/propidium iodide (PI) (Annexin V-FITC/PI) was adopted to detect the apoptosis after EMO treatment, and the Western blot (WB) method was used with the purpose of exploring the changes in protein expression levels of PARP, Bcl-2, and p53 in the cells after treatment. It was found that compared with the original U-Net model, the introduction of the BN layer and the dropout layer can improve the robustness of the U-Net model, and the optimized U-Net model had the highest dice similarity coefficient (DSC) (98.45%) and mean average precision (MAP) (0.88) for the liver tumor segmentation.

## 1. Introduction

Primary liver cancer is currently one of the common malignant tumors with high morbidity and mortality, which has seriously threatened the safety of human life [1]. Surgical treatment is currently the most direct and thorough method for liver treatment, but precise surgical treatment is required to preserve the integrity of the unaffected area of the liver to the greatest extent [2]. The prerequisite for doctors to perform accurate diagnosis and treatment of liver cancer is to accurately segment the lesion area from the patient's imaging treatment. The current manual segmentation method has the highest accuracy, but it will waste a lot of time and energy in the face of massive medical imaging data. In addition, the manual segmentation has the characteristics of non-repeatability and subjectivity [3, 4]. To improve the efficiency of medical image processing and realize the intelligence and repeatability of image segmentation, a large number of experts and scholars have introduced the intelligent algorithms to achieve this goal. At present, the algorithms commonly used for the image segmentation include the support vector machines (SVMs), convolutional neural networks (CNNs), and U-Net [5–7]. Among them, the U-Net model is mainly used for the segmentation of medical images and can fuse the image features of different scales, so it is widely used in the segmentation of medical images [8]. However, the depth of the original U-Net model is not enough to obtain a good network model through fast training. Therefore, to solve this problem, an improvement on the structure of the U-Net was explored in this study.

The article "Automatic Segmentation of Magnetic Resonance Images of Severe Patients with Advanced Liver Cancer and the Molecular Mechanism of Emodin-Induced Apoptosis of HepG2 Cells under the Deep Learning" was published in 2022. Journal: J Healthc Eng.

Surgical resection is limited to the treatment of patients with liver cancer in the early stage, but the patients with advanced liver cancer with the characteristics of fast development and easy metastasis can only inhibit the development of liver cancer through chemotherapy or radiotherapy [9]. Radiotherapy can cause vomiting and gastrointestinal mucosal damage in patients, and doxorubicin and other drugs commonly used in chemotherapy have certain toxicity, which can affect the growth of normal cells in the patient's body [10, 11]. Studies have proved that natural secondary metabolites derived from animals, plants, or microorganisms can reduce the toxic and side effects caused by radiotherapy or chemotherapy and have the advantages of high safety performance and resistance to drug resistance [12]. At present, EMO can intervene in the process of liver cancer, cervical cancer, prostate cancer, and other cancers. It mainly achieves alleviation of cancer disease process by blocking the cell cycle and inhibiting the cell proliferation [13, 14].

## 2. Methodology

### 2.1. Experimental Materials

The MR imaging data related to the “advanced liver cancer” were obtained from The Cancer Imaging Archive, and the data provided by researchers of Harvard beamandrew machine learning and medical imaging on the GitHub were referred. As a result, a total of 1,526 MR images were obtained to construct the “MR Image Data Set of Advanced Liver Cancer.”

### 2.2. Preprocessing of MR Image

During the process of image data collection, there may be more interference in the image due to the changes in environment and magnetic field [15]. Therefore, to improve the effect of image segmentation, the images had to be normalized and standardized when inputting the MR images into the model.

The article "Automatic Segmentation of Magnetic Resonance Images of Severe Patients with Advanced Liver Cancer and the Molecular Mechanism of Emodin-Induced Apoptosis of HepG2 Cells under the Deep Learning" was published in 2022. Journal: J Healthc Eng.

The (0, 1) normalization method was adopted to process the image pixel matrix, and the mathematical expression of this method was given as follows:

(1) $$\begin{array}{c} x^{∼}=\text{Factor}\cdot \frac{x-x_{\min}}{x_{\max}-x_{\min}}. \end{array}$$

In the above equation, *x* was the pixel of input image, *x*_max_ represented the maximum value in the pixel matrix, *x*_min_ represented the minimum value in the pixel matrix, and Factor indicated the normalization coefficient. When it was normalized to (0, 1), then Factor = 1; when it was normalized to (0, 200), then the Factor = 200.

Z score was adopted for the standardization of the MR image, and the mathematical expression of this method was given as follows:

(2) $$\begin{array}{c} x^{\prime }=\frac{x-\bar{x}}{\sigma }. \end{array}$$

In the above equation, $\bar{x}$ represented the average value of the pixel matrix of the inputted image and *σ* represented the standard deviation of the pixel matrix of the inputted image.

The number of MR image data collected in this study was limited by time, cases, and other factors, and the use of deep learning technology for image segmentation required a large amount of data for model training, so it was hoped to expand the original MR samples in the form of data enhancement. The methods commonly used for image data enhancement include flip, random crop, color jittering, shift, scale, contract, noise, rotation, and reflection [16], and the Python was used for data enhancement of the MR images from the third-party database Augmentor.

### 2.3. Design and Improvement of U-Net

U-Net was a network algorithm of the medical cell segmentation proposed by Olaf et al. in 2015. The basic structure of the network is shown in Figure 1. It can be seen that the original U-Net presented a structure similar to the “U,” which contained a total of 23 convolutional layers, 4 downsampling operations, and 4 upsampling operations. Compared with the CNN, there was no fully connected layer in the U-Net. Each execution of downsampling included 2 convolution operations with a convolution kernel size of 3*∗*3 and 1 pooling operation with a size of 2*∗*2, while the upsampling operation only included 2 convolution operations with a convolution kernel size of 3*∗*3, and finally, a convolution layer with a convolution kernel size of 1*∗*1 was added to the U-Net.

Based on the original structure of U-Net, the BN layer and the dropout layer were added to improve the structure of the model, and the hyperparameters of the model were adjusted to improve the robustness of the model.

It can be observed from Figure 2(a) that when the traditional neural network was adopted for standardization, the sample data were standardized before the samples were inputted into the network, which reduced the difference among the inputted samples. From Figure 2(b), it can be known that the batch normalization [17] standardized the inputted data of each hidden layer based on the standardization results of traditional neural network. After the effect of activation function ReLU, the output of the first hidden layer was *L*_1_ = *ReLU*(*W*_*L*1_ + *B*_*L*1_). In the calculation of the hidden layer standardized by the batch normalization, it was necessary to process the matrix *x* of the input data using the linear transformation to obtain the input value *q*_1_ in the hidden layer. Secondly, *q*_1_ was standardized, and the average *μ*_*y*_ and standard deviation $\sqrt{\sigma_{y}^{2}+\varepsilon }$ were subtracted to obtain the output value *q*_2_. *μ*_*y*_ is referred to the average value of the selected batch, and *μ*_*y*_=1/*m*∑_*i*=0_^*m*^*W*_*L*_1_*x*_1__. The standard deviation was also the standard deviation of a specific batch, and *σ*_*y*_^2^=1/*m*∑_*i*=0_^*m*^(*W*_*L*_1_*x*_1__ − *μ*_*y*_)^2^ to prevent errors when *σ*_*y*_^2^=0. The processed *q*_2_ data showed a normal distribution characteristic, which reduced the expressive ability of the network model, so new parameters (*m* and *B*) had to be introduced. *m* and *B* were obtained by self-learning of the network after training, *q*_3_ can be obtained after data *q*_2_ were processed with the introduced parameters, and the output *L*_1_ of the hidden layer was obtained using the activation function ReLU.

The article "Automatic Segmentation of Magnetic Resonance Images of Severe Patients with Advanced Liver Cancer and the Molecular Mechanism of Emodin-Induced Apoptosis of HepG2 Cells under the Deep Learning" was published in 2022. Journal: J Healthc Eng.

The basic structure parameters of the U-Net optimized in this study are shown in Table 1.

Finally, the U-Net model was built and tested under the Keras deep learning framework. The process of segmenting the MR image of liver cancer patients using the optimized U-Net model is shown in Figure 3.

### 2.4. Evaluation Indexes of Liver Tumor Segmentation Efficacy

The DSC and recall and precision (R-P) were utilized to evaluate the segmentation efficacy of liver tumor by the optimized U-Net. Among them, DSC was used for evaluating the degree of overlap between the segmented tumor and the gold standard tumor. The closer it was to 1, the more similar the segmentation result was to the gold standard result. The calculation equation can be written as follows:

(3) $$\begin{array}{c} \text{DSC}\left(T,P\right)=\frac{2\left|T\cap P\right|}{\left|T\right|+\left|P\right|}. \end{array}$$

In the above equation, *T* was the true value and *P* was the prediction value outputted by the model.

Recall was used to evaluate the correct rate of image classification. The closer it was to 1, the better the classification effect. The calculation equation was given as follows:

(4) $$\begin{array}{c} \text{recall}=\frac{TP}{TP+FN}. \end{array}$$

In the above equation, *TP* is referred to the truth-positive value (both the classification result and the gold standard result were positive samples) and *FN* is referred to the false-negative value (the positive samples were predicted as negative samples).

The article "Automatic Segmentation of Magnetic Resonance Images of Severe Patients with Advanced Liver Cancer and the Molecular Mechanism of Emodin-Induced Apoptosis of HepG2 Cells under the Deep Learning" was published in 2022. Journal: J Healthc Eng.

Precision was to evaluate the error rate of wrong classification of the samples. The closer it was to 1, the better the classification effect, and it can be calculated with the following equation:

(5) $$\begin{array}{c} \text{precision}=\frac{TP}{TP+FP}. \end{array}$$

In the above equation, the *FP* is referred to the false-positive value (the negative samples were predicated as the positive samples).

### 2.5. Test on Cell Viability of HepG2 after EMO Treatment

Studies had shown that plants can selectively enrich the growth-promoting bacteria Stenotrophomonas through roots and then promote the accumulation of EMO in the roots (as shown in Figure 4) [18]. Studies had also shown that EMO can inhibit the proliferation of cancer cell through cell cycle arrest, autophagy, and apoptosis [19].

Based on this, the changes in cell viability by different concentrations of EMO (0 *μ*mol/L, 10 *μ*mol/L, 20 *μ*mol/L, 40 *μ*mol/L, 60 *μ*mol/L, 80 *μ*mol/L, and 100 *μ*mol/L) effecting on HepG2 cells at the 0th, 12th, 24th, 26th, and 48th hour were compared. The activity of cell mitochondrial dehydrogenase was tested by MTT. Firstly, the cells in the logarithmic growth phase were collected and inoculated in a 96-well plate after the cell density was adjusted to 1 × 10^4^ for cultivation overnight; each well was supplemented with 10 *μ*L of different concentrations of EMO (each concentration was added for 3 wells), respectively, and then incubated for 24 hours after mixing fully; the medium was discarded, and 100 *μ*L of 5 mg/mL MTT was added to each well, shaken, and mixed at low speed for around 10 minutes; the absorbance of each well was detected at 560 nm wavelength with a microplate reader, and finally, the results were displayed by IC50 (the concentration at which cell viability was inhibited by 50%).

### 2.6. Test on Cell Morphology of HepG2 after EMO Treatment

After adjusting the cell density to 1 × 10^5^, the cells were inoculated in a 12-well plate for cultivation overnight; each well was supplemented with 10 *μ*L of 10 *μ*mol/L (low concentration), 40 *μ*mol/L (medium concentration), and 80 *μ*mol/L (high concentration) EMO (each concentration was added for 3 wells), respectively, and then incubated for 24 hours after mixing fully. The morphologies of HepG2 cells treated with different concentrations of EMO and untreated (control group) were observed with a light-induced microscope (Olympus, Japan), and related pictures should be taken.

The article "Automatic Segmentation of Magnetic Resonance Images of Severe Patients with Advanced Liver Cancer and the Molecular Mechanism of Emodin-Induced Apoptosis of HepG2 Cells under the Deep Learning" was published in 2022. Journal: J Healthc Eng.

### 2.7. Detection on Apoptosis of HepG2 after the EMO Treatment

AO combined with EB was adopted to stain the HepG2 in the control group, low concentration, medium concentration, and high concentration EMO treatment for 16 hours. The cells were rinsed with phosphate-buffered saline (PBS) twice before adding the dyes, and 50 *μ*g/mL mixed dyes made of 100 *μ*g/mL AO and 100 *μ*g/mL EB at the ratio of 1 : 1 were added to each well, so that the cells were completely immersed in the solution, and then, they were immediately placed under a fluorescent inverted microscope (Olympus, Japan) to observe the luminous state of the cells, and related pictures should be taken.

The Annexin V-FITC/PI Cell Apoptosis Kit was used for the qualitative and quantitative analysis of the cells in the control group and the treatment groups with EMO with different concentrations. Firstly, the cells in different treatment groups were prepared to single-cell suspensions of 1 × 10^6^ cells/mL with PBS, placed in a low-temperature centrifuge after adding 1 mL of the suspension, and centrifuged at 1,000 rpm for about 10 minutes at the temperature of 4°C to collect the precipitate; the above steps were repeated for three times; the cells were resuspended with 500 *μ*L binding solution and mixed fully after adding 10 *μ*L of Annexin V-FITC reagent and 5 *μ*L of PI reagent to react in a dark box at the room temperature lasting for 20 minutes; Annexin V-FITC and PI fluorescence were detected with a flow cytometer (Thermo Fisher Scientific, USA) at the wavelengths of 488 nm–630 nm, respectively.

### 2.8. Detection on Levels of Related Proteins in HepG2 after Treatment with EMO

The radio-immunoprecipitation assay (RIPA) cell lysate was used for cell lysis on ice, and then, the cells were centrifuged, and the cell protein supernatant was collected. The protein concentration was detected using the bicinchoninic acid (BCA) protein quantification kit. The separate gels and concentrated gels of different concentrations were prepared according to the molecular weights of the target protein and up-sampled in the sample holes, and then, the electrophoresis was performed at 80 V and then 120 V, respectively, until the bromophenol blue dye solution was 1 cm from the bottom of the gel. The gels were cut and transferred with polyvinylidene fluoride (PVDF) membrane. The transferred PVDF membrane was placed in a blocking solution for 60 minutes and rinsed with the blocking solution three times and then incubated with the poly ADP-ribose polymerase (PARP), Bcl-2, and p53 primary antibody overnight at a temperature of 4°C. It was rinsed with the blocking solution another three times and then incubated with corresponding secondary antibody for around 120 min at the condition of room temperature; the enhanced chemiluminescence (ECL) color developing solution was supplemented to develop in the gel imaging system (Bio-Rad, USA). Quantity One was used for image acquisition and gray value analysis.

The article "Automatic Segmentation of Magnetic Resonance Images of Severe Patients with Advanced Liver Cancer and the Molecular Mechanism of Emodin-Induced Apoptosis of HepG2 Cells under the Deep Learning" was published in 2022. Journal: J Healthc Eng.

### 2.9. Statistical Analysis

GraphPad was used for data processing, and the one-way ANOVA process in SPSS 19.0 was used for analysis. The experimental data of the mechanism of EMO on the apoptosis of HepG2 cells were all expressed as mean ± standard deviation, and Duncan's multiple comparisons were used to analyze the differences between groups. It was considered that *P* < 0.05 indicated that the difference was statistically significant, *P* < 0.05 indicated there was a significant difference, and *P* < 0.01 indicated there was an obviously great difference.

## 3. Results and Discussion

### 3.1. Performance Test of Optimized U-Net

The performance of the U-Net model with and without the BN layer was compared, and the results are given in Figure 5. It can be seen that as the number of training increased, the DSC value of the U-Net model without the BN layer showed a decreasing trend, indicating that the model training was not successful. This may be because the U-Net model used the random parameter initialization. Similar to other research results, adding BN layer to FCN model can improve the efficiency and accuracy of brain image segmentation [20].

The test results of U-Net adding with and without the dropout layer were compared optimized by the batch gradient descent (BGD), stochastic gradient descent (SGD), Newton's method (NM), quasi-newton method (QNM), conjugate gradient (CG), and Adam optimization algorithms, and the results were given as below. It can be seen from Figures 6(a) and 6(b) that the U-Net model optimized by SGD had the fastest convergence speed and the highest DSC value after stability regardless of whether a dropout layer was added to the U-Net model. Taking the result of SGD optimization as an example, it was found based on the comparison that the test result of the U-Net model with the dropout layer was remarkably better than the model without the dropout layer, and the DCS value was increased by about 2.24%. It shows that adding a dropout layer can prevent the model from overfitting or generalization, and it also improves the segmentation ability and robustness of the model [21].

Finally, the changes in training DSC value of the improved U-Net model before and after the enhancement of the MR image data were compared. It can be observed from Figure 7 that the convergence speed of the model after the data enhancement was faster than that before the data enhancement greatly, and with the gradual increase in the number of iterations, the model became stable gradually. When the maximum number of iterations was reached, the DSC verification result of the model after data enhancement was 97.8%, while the DSC verification result of the model before the data enhancement was 94.55%, so it increased by 3.25%.

The article "Automatic Segmentation of Magnetic Resonance Images of Severe Patients with Advanced Liver Cancer and the Molecular Mechanism of Emodin-Induced Apoptosis of HepG2 Cells under the Deep Learning" was published in 2022. Journal: J Healthc Eng.

### 3.2. Segmentation Efficacy of MR Liver Tumor Based on the Optimized U-Net Model

The application effects in liver tumor segmentation of original U-Net, convolutional neural network (CNN), FCN, regional growth (RG), and Snakes were compared with the effect of the optimized U-Net algorithm in this study, and the results are shown in Figure 8. It can be seen from Figure 9(a) that the segmentation efficacy of U-Net, CNN, FCN, and the improved U-Net model was similar to the gold standard segmentation efficacy, while that of RG was excessively segmented when the distinction between liver tumors and surrounding tissues was not high. Under the condition of uneven grayscale distribution of MR images and uneven surface of the tumor, under segmentation could be found for the Snakes. The segmentation efficacies of different models were quantitatively compared, and recall and precision values were used to draw the P-R curve to obtain the area under the PR curve mAP. From Figure 9(b), it can be seen that the improved U-Net model had the highest mAP value (0.88), followed by the original U-Net model (0.74), while the Snakes model had the smallest mAP value (0.53).

### 3.3. Impacts of EMO on Cell Viability and Proliferation of HepG2

The MTT was used to determine the effect of different concentrations of EMO on the viability of HepG2 cells. It can be seen from Figure 9(a) that with the gradual increase in treatment time, the viability of HepG2 cells gradually decreased after treatment with different concentrations of EMO. It meant that the higher the EMO concentration, the lower the viability of HepG2 cells. The blue-purple formazan crystal staining was adopted to observe the changes in the number of HepG2 viable cells after treatment with different concentrations of EMO. It can be known from Figure 9(b) that the formation of formazan crystals was proportional to the number of viable cells. With the gradual increase in EMO concentration, the amount of formazan crystal gradually decreased, which was consistent with the test results of cell viability.

### 3.4. Impacts of EMO on Morphology and Staining Results of HepG2

First, the changes in cell morphology, AO/EB, and DAPI staining results of HepG2 cells treated with different concentrations of EMO were observed under a microscope. The results are shown in Figure 10. It can be seen that the HepG2 cells treated with 0 *μ*mol/L EMO were tightly connected and exhibited the irregular spindle shapes. With the increasing concentration of EMO, the cell outline became blurred, most of the cells came off, and the number of adherent cells decreased, similar to the characteristics of apoptosis. The AO/EB was used for cell staining, and it can be seen that as the concentration of EMO increased, the proportion of green fluorescence in HepG2 cells gradually decreased, while the proportion of orange-red fluorescence gradually increased; when the EMO concentration reached 100 *μ*mol/L, HepG2 cells all became red. The results of DAPI staining showed that with the gradual increase in EMO concentration, the blue fluorescence in HepG2 cells gradually decreased, showing a dose-dependent manner.

The article "Automatic Segmentation of Magnetic Resonance Images of Severe Patients with Advanced Liver Cancer and the Molecular Mechanism of Emodin-Induced Apoptosis of HepG2 Cells under the Deep Learning" was published in 2022. Journal: J Healthc Eng.

## 4. Conclusion

To improve the effect of deep learning algorithm in tumor segmentation in images and to explore the molecular mechanism of the impacts of EMO on liver cell apoptosis, the U-Net model was optimized in this study to segment the MR images of liver cancer patients. It was found that the improved U-Net model can improve the efficiency and robustness of tumor segmentation, and the segmentation effect was significantly higher than other advanced models.

## Figures and Tables

**Figure 1:** Basic structure of U-Net.

**Figure 2:** Normalization flows of traditional and batch.

**Figure 3:** Process of segmenting the MR image of liver cancer patients using the optimized U-Net network.

**Figure 4:** Accumulation of EMO in plant roots.

**Figure 5:** Impacts of the BN layer on test results of the U-Net.

**Figure 6:** Impacts of dropout layer optimized by various algorithms on the test results of U-Net model.

**Figure 7:** Test results of U-Net model before and after the data enhancement.

**Figure 8:** Analysis on segmentation efficacy of liver tumor with different models.

**Figure 9:** Impacts of different concentrations of EMO on cell viability of HepG2.

**Figure 10:** Morphology and staining results of HepG2 after being treated with EMO in different concentrations.

**Table 1:** Structure parameters of optimized U-Net model.

Layer no.	Structure
1	Batch_Nor 1
2-1	Conv 1–32
2-2	Conv 1–32
3	Maxpooling 1
4	Batch_Nor 2
5	Dropout (0.1)
6-1	Conv 2–64
6-2	Conv 2–64
7	Maxpooling 2
8	Batch_Nor 3
9	Dropout (0.1)
10-1	Conv 3–128
10-2	Conv 3–128
11	Maxpooling 3
12	Batch_Nor 4
13	Dropout (0.2)
14-1	Conv 4–256
14-2	Conv 4–256
15	Maxpooling 4
16	Batch_Nor 5
17	Dropout (0.2)
18-1	Conv 5–512
18-2	Conv 5–512
19	Maxpooling 5
20	Batch_Nor 6
21	Dropout (0.3)
22	Upsampling + merge 1
23	Batch_Nor 7
24	Dropout (0.2)
25-1	Conv 6–256
25-2	Conv 6–256
26	Upsampling + merge 2
27	Batch_Nor 8
28	Dropout (0.2)
29-1	Conv 7–128
29-2	Conv 7–128
30	Up-sampling + merge 3
31	Batch_Nor 9
32	Dropout (0.1)
33-1	Conv 8–64
33-2	Conv 8–64
34	Upsampling + merge 4
35	Batch_Nor 10
36	Dropout (0.1)
37-1	Conv 9–32
37-2	Conv 9–32
38	Conv 10-1

The article "Automatic Segmentation of Magnetic Resonance Images of Severe Patients with Advanced Liver Cancer and the Molecular Mechanism of Emodin-Induced Apoptosis of HepG2 Cells under the Deep Learning" was published in 2022. Journal: J Healthc Eng.

## Data Availability

The dataset used in this study is available from the corresponding author upon request.
